This article has been retracted.

# Lithium treatment extends human lifespan: findings from the UK Biobank

**DOI:** 10.18632/aging.204476

**Published:** 2023-01-11

**Authors:** Elisa Araldi, Catherine R. Jutzeler, Michael Ristow

**Affiliations:** 1 Energy Metabolism Laboratory, Institute of Translational Medicine, Swiss Federal Institute of Technology (ETH) Zürich, Schwerzenbach CH-8603, Switzerland; 2 Center for Thrombosis and Hemostasis and Preventive Cardiology and Preventive Medicine, Center for Cardiology, University Medical Center of the Johannes Gutenberg University Mainz, Mainz D-55131, Germany; 3 Biomedical Data Science Lab, Institute of Translational Medicine, Swiss Federal Institute of Technology (ETH) Zürich, Zürich CH-8008, Switzerland; 4 Institute of Experimental Endocrinology and Diabetology, Charité Universitätsmedizin Berlin, Berlin D-10117, Germany

**Keywords:** geroprotection, human, nutrition, pharmacology, psychiatry

## Abstract

Lithium is a nutritional trace element that is also used pharmacologically for the management of bipolar and related psychiatric disorders. Recent studies have shown that lithium supplementation can extend health and lifespan in different animal models. Moreover, nutritional lithium uptake from drinking water was repeatedly found to be positively correlated with human longevity. By analyzing a large observational aging cohort (UK Biobank, *n* = 501,461 individuals) along with prescription data derived from the National Health Services (NHS), we here find therapeutic supplementation of lithium linked to decreased mortality (*p* = 0.0017) of individuals diagnosed with affective disorders. Subsequent multivariate survival analyses reveal lithium to be the strongest factor in regards to increased survival effects (hazard ratio = 0.274 [0.119–0.634 CI 95%, *p* = 0.0023]), corresponding to 3.641 times lower (95% CI 1.577–8.407) chances of dying at a given age for lithium users compared to users of other anti-psychotic drugs. While these results may further support the use of lithium as a geroprotective supplement, it should be noted that doses applied within the UK Biobank/NHS setting require close supervision by qualified medical professionals.

## INTRODUCTION

The trace element lithium is a naturally occurring alkali metal. Owing to its mood-stabilizing properties [1, 2], lithium has been prescribed for more than 50 years to individuals affected by mood and affective disorders.

Lithium is the most effective maintenance treatment for bipolar disorders [3, 4] and alone or in conjunction with other psychotropic drugs, it can be used as an acute therapy for other mood and affective disorders (ICD10 F30-39), such as acute mania and bipolar depression [5, 6]. Since lithium requires constant monitoring to ensure that its plasma concentration is maintained between target clinical concentrations of 0.4-1mmol, in the current clinical UK guidelines for affective disorders [3], lithium is not recommended as the first-line acute treatment to mania or hypomania, while other anti-psychotic medications are preferred. While lithium efficacy in relieving affective disorders long-term and preventing suicides is well established [7], recent studies both in animal models and in humans have uncovered that lithium may have life-extending properties.

Lithium increases longevity in the nematode *Caenorhabditis elegans*, both at clinical concentrations [8] and in trace amounts [9], in the fruit fly *Drosophila melanogaster* [10], as well as in yeast (*Schizosaccharomyces pombe*) [11]. In *Drosophila*, lithium increases lifespan by inhibiting glycogen synthase kinase-3 (GSK-3) and activating nuclear factor erythroid 2-related factor (NRF-2) [10], suggesting that lithium regulates metabolism and stress resistance. When administered to mice, lithium given at concentrations comparable to the therapeutic ranges for the treatment of human bipolar disorder improves metabolic parameters without significantly extending lifespan [12, 13]. The broad effects of lithium on lifespan in several model organisms suggest that it exerts evolutionary conserved mechanisms to promote healthy aging.

Nutritionally ingested lithium, as present in plant-derived foods and drinking water, is readily bioavailable and evenly disseminated in every tissue, but its distribution in food and water is variable and region-dependent [14, 15]. Using geographic differences in lithium concentration as a natural experiment, studies in independent populations worldwide have demonstrated a positive correlation between trace amounts of lithium in drinking water and longevity [9, 16, 17]. The protective effects of higher dose of lithium intake on all-cause mortality have indirectly been evaluated in prospective intervention studies aimed at comparing the clinical efficacy and suicide rates of lithium on patients suffering from bipolar and related disorders [18, 19]. While highly informative, these studies include mostly middle-aged individuals (43.78 ± 12.94 years) and, more importantly, have a rather short intervention/observation period (2.52 ± 1.05 years). The demographics and observation time of these studies are therefore suboptimal to capture the life-extending properties of lithium in the aging population. In addition, accidental causes of deaths were not excluded from most of these studies potentially confounding the findings. Addressing these shortcomings, we leveraged data from the UK Biobank [20], a large well-characterized and long-term observational population cohort where age of recruitment is 56.41 + 8.09 years and follow-up time is 11.90 ± 1.24 years, to provide interventional evidence that lithium increases lifespan in humans.

## RESULTS

Mood disorders, which are classified in the International Statistical Classification of Diseases and Related Health Problems (10th Edition) (ICD10) with diagnosis codes F30-F39 (onwards globally referred to as F3X) [21], are disturbances of affect or mood and often lead to depression or elation. In the highly characterized and healthcare-linked UK Biobank cohort, we have analyzed National Health Services (NHS) clinical records of participants to identify individuals with at least one ICD10-defined F3X mood affective disorder diagnosis since 1990. F3X-diagnosed individuals constitute a demographics that is significantly different from the rest of the UK Biobank cohort: they are older, have a higher suicide rate, are more frequently affected by comorbidities such as diabetes, cardiovascular diseases and cancer (Table 1 [excluding suicides], Supplementary Table 1 [including suicides]), and, importantly, have a significantly lower lifespan than controls (Figure 1A, Supplementary Figure 1A). A Cox proportional hazard model shows that F3X diagnoses significantly contribute to shortened lifespan (Figure 1B, Supplementary Figure 1B). Analysis of the causes of death indicates that F3X-diagnosed individuals are more likely to die due to suicides, respiratory diseases, mental disorders, diseases of the nervous system, as well as COVID-19, while they are less likely to succumb from cancer (Supplementary Table 2).

**Table 1:** Baseline characteristics, morbidities, and physical or lifestyle traits of individuals with or without ICD10-defined F3X affective disorders diagnoses in NHS clinical records since 01.01.1990.

**Baseline characteristics**	**Control (*n* = 348049)**	**Users diagnosed with F3X (*n* = 62129)**	***p*-value**
Age at recruitment [years]^*^	56.68 ± 8.05	54.93 ± 8.14	0.00E+00
Sex (male) [%] (counts)	47.02 (163660)	34.32 (21325)	0.00E+00
Deaths [%] (counts)	3.29 (11451)	3.53 (2195)	1.95E-03
Age at Death [years]^*^	70.63 ± 7.14	69.91 ± 7.42	1.63E-05
**Morbidities**			
Diabetes [%] (counts)	4.79 (16599)	6.30 (3888)	3.07E-56
Cancer [%] (counts)	7.27 (25161)	8.07 (4981)	1.83E-12
Fractured bones in last 5 years [%] (counts)	9.06 (31308)	11.42 (7030)	4.25E-76
Other serious medical condition/disability [%] (counts)	18.61 (63563)	26.94 (16173)	0.00E+00
Cardiovascular disease [%] (counts)	28.79 (99782)	31.27 (19321)	6.97E-36
Blood clots, DVT, bronchitis and emphysema [%] (counts)	3.64 (12632)	5.36 (3311)	2.97E-91
**Traits**			
Townsend deprivation index^*^	−1.41 ± 3.01	−0.85 ± 3.25	0.00E+00
Sleep duration [hours]^*^	7.15 ± 1.06	7.13 ± 1.32	3.62E-08
Smoking [PackYears]^*^	7.45 ± 14.74	9.98 ± 16.82	2.47E-275
Physical exercise [Summed MET minutes/ week]^*^	2688.64 ± 2715.85	2586.73 ± 2758.85	2.86E-14
Alcohol intake [weekly units]^*^	7.48 ± 8.86	6.62 ± 9.48	3.17E-107
BMI [kg/m^2^]	27.26 ± 4.64	28.09 ± 5.36	0.00E+00

Suicides are excluded from the dataset. ^*^Denotes mean ± standard deviation; *p*-values are obtained with two-tailed t-test for quantitative data and with chi-squared contingency test for categorical data. Abbreviations: DVT: deep vein thrombosis; BMI: body mass index; MET: metabolic equivalent of task.

**Figure 1:** **Individuals with F3X diagnoses have shorter lifespan.** (**A**) Kaplan-Meier curve of survival probability in individuals with or without ICD10-defined F3X affective disorders diagnoses in NHS clinical records since 01.01.1990. Suicides are excluded from the dataset; *p*-value of the logrank test is reported. (**B**) Forest Plot of Cox proportional hazard multivariable modeling on overall survival in individuals with or without ICD10-defined F3X affective disorders diagnoses in NHS clinical records since 01.01.1990. Suicides are excluded from the dataset. Abbreviations: DVT: deep vein thrombosis; BMI: body mass index.

Due to the detrimental and diagnosis-specific effects on lifespan of individuals with mood and affective disorders, and considering that all the patients that take lithium must have at least one F3X diagnosis, we evaluated differences in survival in individuals with F3X diagnoses that are either taking lithium or other psychotropic medications (Figure 2A). By analyzing NHS prescription data, we selected individuals that had taken either lithium, in the therapeutic formulation of lithium carbonate (including brand name equivalent compounds Priadel™, Camcolit™, and Liskorum™), or other anti-psychotic drugs (Supplementary Figure 2) for at least three consecutive months and within 6 months of the time of last recorded event (either death, or at the date of last censoring) (Figure 2A). Patients prescribed with lithium took the drug on average longer than individuals prescribed other anti-psychotic medications, had a longer interval between the first and last F3X diagnoses, and had more cumulative F3X episodes (Supplementary Figure 3B, 3C, 3E, 3F), while the age at onset of the diagnosis and episodes per year were unchanged (Supplementary Figure 3A–3D, 3F). These data support the current UK indications for lithium use in mood affective disorders [3]. Among the 348 lithium users, there were no suicide deaths, while in 1717 users of other psychotic drugs there were 5 deaths by suicides (Supplementary Table 3). Since deaths by suicides were not present among lithium treated individuals, only deaths not caused by accident nor self-inflicted causes were considered in subsequent analyses.

**Figure 2:** **Study design to assess the effects of lithium on longevity in the UK Biobank.** (**A**) Flowchart for inclusion and exclusion criteria in the UK Biobank cohort. Diagnoses and prescriptions were retrieved from GP clinical records and primary care datasets in National Health Service (NHS) records. One lithium user was matched to two other anti-psychotic drug users with propensity score matching using a nearest neighbor distance algorithm and the parameters indicated. (**B**) Most frequent ICD10 F3X diagnoses in the matched cohort of lithium and other anti-psychotic drug users.

To ensure that the outcomes of lithium use on survival were not affected by confounding variables, such as baseline population characteristics, we used propensity score matching with nearest neighbor distance algorithm (Figure 2A) [22]. Propensity score matching (PSM) is a statistical matching method that allows to analyze an observational non-randomized study so that it mimics a randomized controlled trial in a *post-hoc* fashion [23, 24]. While in randomized control trials the propensity score, or probability to assign a treatment based on observed baseline covariates, is defined by the study design, in observational studies PSM allows to selected *a posteriori* individuals to include in control groups based on a distance algorithm that equalizes the values of a defined set of covariates in the treatment group [22]. In the current study, participants using lithium were outnumbered by users of other anti-psychotic drugs, therefore each lithium user was matched to two users of other anti-psychotic drugs for baseline traits including sex, age at recruitment, most common F3X diagnoses, other comorbidities and age at first treatment as a proxy of the length of treatment (Figure 2A). The resulting matched cohorts, composed of 276 lithium users and 552 users of other psychotropic medications, had identical distribution of the 5 most frequent F3X diagnoses (Figure 2B) and baseline characteristics (Table 2). By applying this widely used approach, we ensured that individuals in both groups were comparable in terms of comorbidities, F3X diagnoses, and length of drug use, and therefore the effects on lifespan mediated by the two treatment regimens could be compared excluding confounding effects [23, 24].

**Table 2:** Baseline characteristics, morbidities, most frequent ICD10 F3X diagnoses, and physical or lifestyle traits of in individuals with ICD10-defined F3X affective disorders diagnoses taking lithium and matched subjects prescribed other anti-psychotic medications.

**Baseline characteristics**	**Lithium users (*n* = 276)**	**Other anti-psychotic drug users (*n* = 552)**	***p*-value**
Age at recruitment [years]^*^	57.58 ± 7.51	56.91 ± 7.65	0.2339
Sex (male) [%] (counts)	40.94 (113)	38.95 (215)	0.5805
Deaths [%] (counts)	4.35 (12)	10.51 (58)	0.0027
Age at Death [years]^*^	71.49 ± 4.93	70.87 ± 6.28	0.7516
**Medication use**			
Age at first drug use [years]^*^	53.08 ± 10.71	53.80 ± 11.61	0.3876
Length of drug use [years]^*^	16.56 ± 8.37	14.93 ± 8.73	0.0105
**ICD10 F3X diagnoses**			
F3X episodes per year (counts)	1.71 ± 3.21	3.03 ± 16.93	0.2016
Hypomania [F300]	39.49 (109)	36.05 (199)	0.3340
Bipolar affective disorder, unspecified [F319]	20.65 (57)	21.01 (116)	0.9038
Severe depressive episode with psychotic symptoms [F323]	6.52 (18)	6.88 (38)	0.8448
Depressive episode, unspecified [F329]	14.86 (41)	17.93 (99)	0.2651
Recurrent depressive disorder, current episode mild [F330]	26.45 (73)	27.17 (150)	0.8246
**Comorbidities**			
Diabetes [%] (counts)	4.71 (13)	4.53 (25)	0.9065
Cancer [%] (counts)	8.70 (24)	8.33 (46)	0.8598
Fractured bones in last 5 years [%] (counts)	7.97 (22)	7.79 (43)	0.9272
Other serious medical condition/disability [%] (counts)	50.00 (138)	49.82 (275)	0.9608
Cardiovascular disease [%] (counts)	23.19 (64)	24.46 (135)	0.6873
Blood clots, DVT, bronchitis and emphysema [%] (counts)	6.16 (17)	5.43 (30)	0.6710
**Traits**			
Townsend deprivation index^*^	−1.05 ± 3.21	−0.83 ± 3.41	0.3668
Sleep duration [hours]^*^	7.47 ± 1.37	7.70 ± 1.55	0.0461
Smoking [Pack Years]^*^	8.50 ± 16.49	8.70 ± 16.20	0.8677
Physical exercise [Summed MET minutes/week]^*^	1971.51 ± 2055.12	2329.64 ± 2697.01	0.0771
Alcohol intake [weekly units]^*^	6.20 ± 8.21	5.35 ± 7.97	0.1538
BMI [kg/m^2^]	27.77 ± 4.67	27.82 ± 4.98	0.8925

Suicides are excluded from the dataset; ^*^denotes mean ± standard deviation. *p*-values are obtained with two-tailed t-test for quantitative data and with chi-squared contingency test for categorical data. Abbreviations: DVT: deep vein thrombosis; BMI: body mass index; MET: metabolic equivalent of task.

Lithium significantly extends the lifespan of its users compared to individuals taking other anti-psychotic medications (Figure 3A). Cox proportional hazard model shows that taking lithium is the covariate that most significantly contributes to increased longevity in the study (Figure 3B), with a logHR of −1.292 (−2.129067 to −0.455455 CI 95%), or hazard ratio of 0.274 (0.119–0.634 CI 95%) corresponding to 3.641 times lower (95% CI 1.577–8.407) chances of dying at a given age for lithium users compared to other anti-psychotic drug users. Characteristics such as male gender, having been diagnosed with diabetes, blood clots or cancer increase the hazard ratio, as previously shown [25, 26]. Interestingly, lithium significantly increases longevity both in males and female, therefore lithium exerts its geroprotective effect independently of sex (logrank female *p*-value: 0.0253; logrank male *p*-value: 0.0315) (Supplementary Figure 4A, 4B). Similar results were obtained when including also the deaths by suicides in the cohort taking other anti-psychotic drugs (Supplementary Figure 5A, 5B, Supplementary Table 4). Overall our data demonstrates in a large population-based aging observational cohort that lithium has life-extending properties. The causes of death between lithium users and other psychotropic drug users were not significantly different (Supplementary Table 5).

**Figure 3:** **Lithium extends lifespan.** (**A**) Kaplan-Meier curve of survival probability in individuals in the cohort described in A. Suicides are excluded from the dataset; p-value of the logrank test is reported; (**B**) Forest Plot of Cox proportional hazard multivariable modeling on overall survival in individuals in the cohort described in A. Suicides are excluded from the analysis. Abbreviations: DVT: deep vein thrombosis; BMI: body mass index.

## DISCUSSION

This study is the first to evaluate the effects of lithium on lifespan in a large aging observational cohort. We have employed a state-of-the-art statistical algorithm, namely propensity score matching, to take advantage of the large amount of observational data in the UK Biobank and simulate a randomized control trial setting to evaluate whether lithium is a geroprotective agent in humans. We have unveiled that lithium at therapeutic concentrations is not only effective in ameliorating mental health, but it is also able to decrease mortality in individuals affected by F3X diagnoses, a demographics that would normally be more fragile and shorter-lived compared to healthy individuals, as also shown in this study. An alternative interpretation for these findings is that lithium in F3X-diagnosed patients has fewer lifespan-decreasing effects than other medications used to treat F3X diagnoses, and therefore it protects its users from side effects which may lead to premature death.

It needs to be noted that lithium is not prescribed in patients unless they suffer from a F3X diagnosis, i.e., there is an indication bias in the selection of individuals included in the analysis. This bias is unavoidable in observational studies, where drugs are administered to participants that have an underlying condition, and only preventable if designing an *ad hoc* clinical trial where effects of lithium on longevity would be evaluated exclusively in healthy individuals. Even considering these limitations, this study unambiguously revealed that lithium is the most significant factor in reducing mortality in patients with affective disorders, and encourages further investigations in healthy individuals.

Our findings are in line with previous works demonstrating that trace amounts of lithium in drinking water are positively correlated with longer lifespan [9, 17] and cognitive improvement [27], and support the idea that lithium could be used as a nutritional longevity supplement [16]. Lithium use in humans has been linked with molecular changes associated with longevity. Long-term lithium-treated bipolar disorder patients are protected from leukocyte telomere shortening [28], and lithium carbonate therapy has been associated with improved kidney function through inhibition of GSK3beta activity and decreased senescence signaling in urinary exfoliated podocytes [29]. In our analyses, due to the relatively limited size of the lithium cohort, we cannot evaluate if specific pathologies are delayed thanks to lithium, and larger cohorts should be used to pinpoint which biological processes mostly contribute to the lithium-mediated lengthening of lifespan in human cohorts. Therefore, the full extent of the molecular mechanisms of lithium-induced longevity in humans still remains elusive and should be further investigated.

## MATERIALS AND METHODS

### Dataset

The UK Biobank is a prospective study that recruited 502,611 participants aged between 38 and 73 years from 22 sites across the UK with baseline measures collected between 2006 and 2010. Data have since been linked to hospital, prescription and mortality records [20]. This research has been conducted using the UK Biobank Resource (Application Number 48008). UK Biobank had obtained ethics approval from the North West Multi-centre Research Ethics Committee (approval number: 11/NW/0382) and had obtained informed consent from all participants.

Clinical and prescription NHS data (primary care GP datasets, data providers TPP - https://www.tpp-uk.com/ and EMIS - https://www.emishealth.com/) were retrieved on 01.10.2021. Codes for lithium and psychotropic medications were obtained from using SNOMED (EMIS dataset), CTV3 and TPP local codes (TPP dataset). The fields from UK Biobank data download used for this analysis were: ‘53-0.0’ Date of Recruitment, ‘21022-0.0’ Age at Recruitment, ‘34-0.0’ Year of birth, ‘52-0.0’ Month of Birth, ‘40007-0.0’ Age at Death, ‘40000-0.0’ Date of Death, ‘40001-0.0’ Cause of Death, ‘31-0.0’ Sex, ‘22009-0.1’ to ‘22009-0.10’ Genetic principal components (PC) 1-10, ‘22040-0.0’ Summed MET minutes per week for all activity, 21001-0.0 BMI, ‘189-0.0’ Townsend deprivation index, ‘20161-0.0’ PackYears, ‘20116-0.0’ Smoking status, ‘1160-0.0’ Sleep duration, ‘2443-0.0’ Diabetes diagnosed by doctor, ‘2453-0.0’ Cancer diagnosed by doctor, ‘2463-0.0’ Fractured/broken bones in last 5 years, ‘2473-0.0’ Other serious medical condition/disability diagnosed by doctor, ‘6150-0.0’ Vascular/heart problems diagnosed by doctor.

### Inclusion/exclusion criteria

Only the participants with clinical data and prescription data were included in the study, under the assumption that the data for the other participants was not available, rather than that these individuals never sought NHS services. Individuals that died of accidental causes (ICD10 codes starting with O, Q, S, T, V, W, Y) were excluded from the analysis. Individuals that had not taken lithium or other anti-psychotic medications for at least 3 consecutive months, and that were not taking these medications within 6 months of the last recorded event (either death or last censoring), were excluded. We used the anatomic therapeutic chemical (ATC) classification system [30] to select the anti-psychotic drugs from the dataset (codes N05A^*^), plus valproic acid (N03AG01). Prescription for lithium carbonate (N05AN01) and brand name formulations (Priadel™, Camcolit™, Liskorum™) were considered as lithium use [19].

### Propensity score matching

Propensity score matching was implemented using logistic regression in scikit-learn [31], Nearest Neighbors unsupervised learner for implementing neighbor searches with 2 neighbors and KDTree algorithm using the following covariates: sex, age at recruitment, most common F3X diagnoses, age at first drug use (as a proxy for length of drug use) and other comorbidities [32–34]. Differences in baseline characteristics of the obtained cohort were calculated with Student’s two-tailed *t*-test for continuous variables or chi-squared two-tailed test using Scipy functions.

### Survival analyses

Since the day of birth is not available for privacy and data protection regulations, the precise age of the participant at the age of recruitment was estimated, taking into account the age between date of birth (DOB) and date of recruitment, assuming that the DOB is on the 15th of the month [35]. This was not the case for 4520 participants, whose birthday was between the beginning of the month and the recruitment date before the 15th of the month. For these participants the estimated age was rounded up to the declared age of recruitment. In the dataset used for these analyses (retrieved on 01.10.2021), 2021-03-20 is the date of the last reported death, therefore that was considered the time of censoring and used to calculate the inferred age of the live participants from the estimated age at recruitment [35]. The inferred age at death was calculated from the estimated age at recruitment and the date of death. The censoring status = 1 indicates that an event occurred (i.e., death), status = 0 indicates that the observation was right censored (i.e., participant was alive the time of censoring, 2021-03-20).

Survival curves were generated with the Lifelines package KaplanMeierFitter function, and *p*-values calculated with logrank test. In Kaplan Meier survival estimates, the survival probability is expressed as proportion of individuals that are alive at that age versus total number of individuals that have died at that age [36].

Multivariate analysis of survival was analyzed with Cox proportional-hazard regression model using Lifelines CoxPHFitter. Proportional hazard assumption was checked with Lifelines function *check_assumption* and it was valid for all covariates. The difference between the age of recruitment and the age of last censoring was the endogenous variable of the model [37], while age at recruitment, sex, genetic principal components 1–20 (as proxy for population ethnic diversity), lifestyle factors, and comorbidities were exogenous variables.

### Data availability statement

Data was obtained through UK Biobank application #48008. The data that supports the findings of this study are available in the supplementary of this article.

All the analyses, figures and tables were created with Python3.7 using the following libraries: pandas v.1.1.4, matplotlib v.3.3.4, seaborn v. 0.11.1, scipy v. 1.4.1, sklearn v.0.0 [31], statsmodels v. 0.11.0, lifelines v.0.25.11, and numpy v.1.19.5 [38].

Custom code for the analyses will be made available at https://github.com/araldi/Lithium-and-survival-in-UKBB.

## Supplementary Materials

Supplementary Figures

Supplementary Tables
